This article has been retracted.

# Mitochondrial Dysfunction Promotes Breast Cancer Cell Migration and Invasion through HIF1α Accumulation via Increased Production of Reactive Oxygen Species

**DOI:** 10.1371/journal.pone.0069485

**Published:** 2013-07-29

**Authors:** Jia Ma, Qing Zhang, Sulian Chen, Binbin Fang, Qingling Yang, Changjie Chen, Lucio Miele, Fazlul H. Sarkar, Jun Xia, Zhiwei Wang

**Affiliations:** 1 Department of Biochemistry and Molecular Biology, Bengbu Medical College, Bengbu, Anhui, China; 2 Department of Orthopedics, The Center Hospital of Bengbu, Anhui, China; 3 Research Center of Clinical Laboratory Science, Bengbu Medical College, Bengbu, Anhui, China; 4 University of Mississippi Cancer Institute, Jackson, Mississippi, United States of America; 5 Department of Pathology and Oncology, Karmanos Cancer Institute, Wayne State University, Detroit, Michigan, United States of America; 6 Department of Pathology, Beth Israel Deaconess Medical Center, Harvard Medical School, Boston, Massachusetts, United States of America; 7 Cyrus Tang Hematology Center, Jiangsu Institute of Hematology, First Affiliated Hospital of Soochow University, Suzhou, Jiangsu, China; University of Illinois at Chicago, United States of America

## Abstract

Although mitochondrial dysfunction has been observed in various types of human cancer cells, the molecular mechanism underlying mitochondrial dysfunction mediated tumorigenesis remains largely elusive. To further explore the function of mitochondria and their involvement in the pathogenic mechanisms of cancer development, mitochondrial dysfunction clones of breast cancer cells were generated by rotenone treatment, a specific inhibitor of mitochondrial electron transport complex I. These clones were verified by mitochondrial respiratory defect measurement. Moreover, those clones exhibited increased reactive oxygen species (ROS), and showed higher migration and invasive behaviors compared with their parental cells. Furthermore, antioxidant N-acetyl cysteine, PEG-catalase, and mito-TEMPO effectively inhibited cell migration and invasion in these clones. Notably, ROS regulated malignant cellular behavior was in part mediated through upregulation of hypoxia-inducible factor-1 α and vascular endothelial growth factor. Our results suggest that mitochondrial dysfunction promotes cancer cell motility partly through HIF1α accumulation mediated via increased production of reactive oxygen species.

## Introduction

Cancer cells display mitochondrial dysfunction to make cells adapt glycolysis to generate ATP even in the presence of oxygen, namely Warburg effect [1]. The mitochondrial dysfunction has been found to be associated with the development of human cancers [2], [3]. It has been reported that mitochondrial dysfunction could be caused by inhibitors of mitochondrial electron transport chain [4], pathogenic mutations in mitochondrial DNA (mtDNA) [3], and mutations in nuclear gene coded electron transport chain proteins [2]. Additionally, accumulating evidence suggests that cancer cells exhibit increased intrinsic reactive oxygen species (ROS) stress partly due to mitochondrial malfunction [5], [6]. The increased ROS in cancer cells may in turn affect certain redoxsensitive molecules and further lead to stimulation of cellular proliferation, cell migration and invasion, contributing to carcinogenesis [7], [8]. However, the underlying molecular mechanisms by which mitochondrial dysfunction increases ROS production and subsequently leads to tumorigenesis are not fully understood.

Emerging evidence suggests that mitochondrial malfunction and hypoxia in the tumor microenvironment are considered as two major factors contributing to the Warburg effect [9], [10]. In solid tumors, hypoxia, which is an oxygen tension below physiologic levels, develops as abnormal proliferation outstrips the blood supply [11]. This hypoxic region is involved in tumor malignancy and proliferation, resulting in the development of resistance to radiotherapy [12]. Hypoxia-inducible factor-1 (HIF-1), a transcription factor that regulates the cellular response to hypoxia, induces several genes that mediate tumorigenesis [13], [14]. It is known that HIF-1 is a heterodimer that consists of the oxygen-sensitive HIF-1α subunit and the constitutively expressed HIF-1β subunit [15], [16]. Under normoxic conditions, HIF-1a is hydroxylated by prolyl hydroxylases on the proline residues in the oxygen-dependent degradation domain [17], [18]. In hypoxic conditions, low oxygen leads to HIF-1α stabilization due to the inhibition of prolyl-hydroxylation and subsequent reduction in HIF-1α ubiquitination and degradation [18].

In addition to the regulation of HIF-1α by oxygen supply, there are also different HIF activators that include growth factors, hormones, cytokines and viral proteins [19]. Interestingly, related observations of ROS regulating HIF-1α expression appear to be controversial. For example, multiple studies have shown that increased HIF-1α expression contributes to mitochondrial activity and ROS formation during hypoxia [20], [21]. However, other studies have demonstrated a decrease in HIF-1α with increasing ROS [22]. Moreover, some studies have shown no effects on mitochondrial ROS [23]. These controversy results suggest that further study is required to investigate the relationship between HIF-1 α and ROS.

In the present study, we treated SKBR3 and 4T1 breast cancer cells by an inhibitor of mitochondrial electron transport complex I, rotenone, for 1–2 weeks to establish mitochondrial dysfunction subclones. Each subclone was confirmed to have mitochondrial dysfunction by measurement of oxygen consumption, glucose uptake, and lactate production. We found that mitochondrial dysfunction subclones had elevated levels of ROS production. We further analyzed (a) whether ROS are required for induction of tumor cell migration and invasion; (b) whether ROS production regulate HIF-1α and vascular endothelial growth factor (VEGF) expression; (c) whether ROS govern tumor cell migration and invasion through the regulation of HIF-1α and VEGF expression. This work provides the molecular insight into the role of ROS in the regulation of breast cancer cell migration and invasion.

## Materials and Methods

### Reagents

Antibody against HIF-1α was purchased from BD Biosciences. Antibodies against VEGF and β-actin were purchased from Santa Cruz Biotechnology. Rotenone, PEG-catalase, and antioxidant N-acetyl cysteine were obtained from Sigma. 2′,7′-Dichlorofluorescein diacetate (CM_2_-DCFHDA) was purchased from Invitrogen. mitoTEMPO was purchased from Enzo Life Sciences. 8 µm pore Transwell inserts and Matrigel were bought from BD Biosciences.

### Cell Culture

SKBR3 and 4T1 breast cancer cells were bought from American Type Culture Collection (Rockville, MD). SKBR3 cells were cultured in DMEM medium supplemented with 10% fetal bovine serum and penicillin (100 units/ml) and streptomycin (100 µg/ml). Murine 4T1 breast cancer cells were cultured in 1640 medium supplemented with 10% fetal bovine serum and penicillin (100 units/ml) and streptomycin (100 µg/ml). The subclone cells used in this study were generated by rotenone treatment as described previously [4]. It is important to note that rotenone was absent after clone generation during the clone studies. Briefly, cells were treated for 24 h with rotenone (100 nmol/L), then cultured in drug-free medium for 48 h. Followed by two more cycles of rotenone treatment, cells were then plated at a density of 200 per dish in drug-free medium to allow the formation of colonies, which caused an increase in superoxide generation measured by flow cytometry. Among these clones, two clones with higher ROS from SKBR3 cells were named as A and B, and two clones with higher ROS from 4T1 cells were marked as C and D for further studies.

### ROS Measurement

Intracellular ROS generation was assessed using 2′,7,-dichlorofluorescein diacetate. Briefly, 1×10^6^ cells were plated on the 6-well plates and incubated with DCFH-DA (10 mmol/L) for 30 min at 37°C. Cells were washed and harvested in Hank’s buffered salt solution (HBSS) and analyzed immediately using a BD FACScan flow cytometer. Data were analyzed as single parameter frequency histogram using cell Quest software (BD Biosciences). Results are presented as mean fluorescence intensity.

### Hydrogen Peroxide Measurement

The cells were lysed in 100 µl lysis buffer supplied by the H_2_O_2_ assay kit (Beyotime Institute of Biotechnology, China) to determine the intracellular H_2_O_2_ concentration. The supernatants were obtained by centrifuging at 12,000×*g* for 10 min. The H_2_O_2_ concentrations were measured with the assay kit according to the manufacturer’s instructions [24]. Briefly, 50 µl sample solution was incubated with 100 µl reaction solution at room temperature for 30 min, and then the absorption at 560 nm was measured. The H_2_O_2_ concentration was calculated by the standard curve made from the standard solutions.

### Mitochondrial Respiratory Defect Measurement

ATP measurements were performed using ATP assay Kit (Beyotime). We also investigated the mitochondrial oxidative phosphorylation contribution on ATP production with the addition of ATP synthase inhibitor, oligomycin, as previously described [25]. Briefly, cells were grown to approximately 80% confluence, and then incubated in DMEM containing the following combinations of substrates and inhibitors: 4.5 mg/ml glucose plus 110 mg/l pyruvate; glucose plus 15 mg/ml of oligomycin. Cells were incubated with 15 mg/ml of oligomycin for 20 min before harvesting. The remaining steps were following the manufacturer’s instructions.

Cellular glucose uptake was measured by incubating cells in glucose-free medium with 0.2 Ci/mL [3H] 2-deoxyglucose (specific activity, 40 Ci/mmol) for 60 minutes. After the cells were washed with ice-cold PBS, the radioactivity in the cell pellets was quantified by liquid scintillation counting. Cellular lactate level was measured under normoxia with lactate assay kit (Biovision) following the manufacturer’s instructions. The absorbance was recorded using a microplate reader at a 570-nm wavelength. The data were normalized to the control group.

### Transwell Migration and Invasion Assays

The migration of breast cancer cells and their subclones was performed using a 24-well transwell chamber (Corning) containing gelatin-coated polycarbonate membrane filter (6.5 mm diameter, 8 µm pore size). 1×10^5^ cells suspended in 100 µl culture medium with 1% FBS were seeded into the upper chamber. The lower chamber contained 600 µl culture medium with 10% FBS as a chemoattractant. After 24 h incubation at 37°C in 5% CO_2_, non-migrated cells were scraped from the upper surface of the membrane with a cotton swab, and migrated cells remaining on the bottom surface were fixed with 4% paraformaldehyde, staining with giemsa and photographed under a microscope at 20 magnification. The numbers of migrated cells were counted under a light microscope in 5 randomly-selected fields for each chamber. The invasion of the cancer cells were performed by the same procedure as in the migration assay except that the chamber filter were coated with matrigel (BD Biosciences) and 5×10^5^ cells were seeded into the upper chamber.

### Wound Healing Assay

2×10^5^ cells were added to each well of 6-well plate and cultured at 37°C in 5% CO_2_ until more than 80% confluent. They were then scratched with a standard 200 µl pipette tip, wounded monolayers were washed twice to remove nonadherent cells and images were captured at 0 h, 24 h and 48 h after wounding using a Nikon Eclipse TE300 microscope and a Nikon Plan Fluor 4×0.13 objective.

### Western Blotting Analysis

Western blotting was performed as previously described [26]. Briefly, cells were lysed with a whole-cell extract buffer (50 mM Tris, 150 mM NaCl, 0.1% sodium dodecylsulfate, 5 mM EDTA, 4 mg/ml glycerophosphate) containing freshly protease inhibitors. Total proteins were collected by centrifugation. The proteins were quantified by BCA protein assay. Twenty-five micrograms of lysate proteins were separated by SDS–PAGE and subsequently transferred to a PVDF membrane. The membranes were blocked with a solution of Tris-buffered saline (TBS), 0.1% Tween-20 (TBS-T) containing 5% nonfat milk. The membranes were incubated overnight at 4°C with primary antibodies against human HIF-1α, VEGF, and β-actin. The membranes were washed with TBS-T, and secondary antibodies were added to the membrane for 1 h at 37°C. Membranes were washed with TBS-T, visualized with ECL reagent (Millipore), and exposed to film.

### RNAi-mediated Inhibition of HIF-1α

The target sequence of HIF-1α was selected [27] as followed: 5′-TACGTTGTGAGTGGTATTATT-3′. The 21 nt target sequence served as the basis for the design of the two complementary 55-mer siRNA template oligonucleotides that were synthesized, annealed, and ligated annealed siRNA template were inserted into the pSilencer 4.1-CMV vecter (Ambion). Briefly, shRNA was designed by using the siRNA software according to the sequence target as follows: Forward oligo, 5′-GAT CCC GTT GTG AGT GGT ATT ATT TTC AAG AGA AAT AAT ACC ACT CAC AAC GTA A-3′, Reverse oligo, 5′-AGC TTT ACG TTG TGA GTG GTA TTA TTT CTC TTG AAA TAA TAC CAC TCA CAA CGG-3′. The double stranded DNA sequence was obtained through annealing after chemosynthesis and was inserted into PsilencerTM4.1-CMV vector. The insert production was transformed into *E. coli* cells. Then the clones were picked and sequenced to verify the inserts. Transient transfection was performed using the Cationic lipid Lipofectamine2000 (Invitrogen) with HIF-1a shRNA vector.

## Results

### Generation of Subclones with Higher ROS

Rotenone has been accepted as a blocker of the electron flow through inhibition of complex I and subsequently causing an increase in the production of superoxide due to electron flow bifurcation [4]. Therefore, we used rotenone to increase superoxide generation which leads to subsequent induction of ROS stress in SKBR3 and 4T1 cells. After three cycles of rotenone treatment, cells were plated in drug-free medium to allow the formation of colonies. After subclones are generated, each 18 subclones from SKBR3 and 4T1 cells were picked to measure ROS level. Among 18 SKBR3 subclones, 15 subclones showed significantly higher ROS production compared to their parental SKBR3 cells, 3 subclones showed almost the same ROS level as their parental SKBR3 cells (data not shown). Among 18 4T1 subclones, 14 subclones have obviously higher ROS production than that of their parental 4T1 cells, and 4 subclones showed no difference in ROS production with their parental 4T1 cells (data not shown). Four clones with highest ROS were selected for further studies. Two SKBR3 cells’ subclones with higher ROS were named A and B (Figure S1A), while C and D subclones were selected from 4T1cells (Figure S1B).

### Subclones Exhibiting Mitochondrial Dysfunction

To determine whether increased ROS affect mitochondrial dysfunction, we performed the mitochondrial respiratory defect measurement. As illustrated in Figure 1A, both A and B clones showed increased in glucose uptake and lactate production compared to their parental SKBR3 cells (Fig. 1A). Moreover, both A and B clones had similar total ATP content compared with the parental SKBR3 cells: however; ATP synthesis sensitive to oligomycin that assumed to be contributed by mitochondrial ATP synthase further decreased in A and B clones compared with parental SKBR3 cells (Fig. 1B). Similar results were found in 4T1 cells (Fig. 1B). These results suggest that up-regulation of glycolysis was sufficient to compensate the decreased ATP generation in the mitochondria.

**Figure 1:** Biochemical characterization of mitochondrial dysfunction of both clones of breast cancer cells. A, Comparison of ATP synthase (left), glucose uptake (middle), and lactate production (right) in SKBR3 cells. *P<0.01 vs SKBR3 cells, **P<0.05 vs SKBR3 cells, #P<0.05 vs SKBR3 cells (n = 3). B, Comparison of ATP synthase (left), glucose uptake (middle), and lactate production (right) in 4T1 cells. *P<0.05 vs 4T1 cells, **P<0.01 vs 4T1 cells, #P<0.05 vs 4T1 cells (n = 3).

### ROS Promoted Cell Motility and Invasion

As ROS have been reported to be involved in tumor metastasis [8], we tested the motility and invasive potential of each subclones. Furthermore, to evaluate whether increased ROS were essential for this process, cells were pretreated with the antioxidant N-acetyl cysteine (NAC) before the Transwell assay and wound healing assay. As we expected, four subclones exhibited greater motility compared to their parental cells. More importantly, these migration capacities were significantly inhibited by NAC (Fig. 2A, 2B). Consistent with these results, we observed that these subclones with higher ROS showed highly invasion capacity, which can be inhibited by NAC (Figure S2). In agreement with the Transwell assay, the wound healing assay showed significantly accelerated wound closure in these subclone cells compared to their parental cells after scratch assay (Fig. 3A, 3B). NAC effectively inhibited the wound closure in these subclones (Fig. 3A, 3B). These results indicated that the aggressive cellular behaviors of subclones might be regulated by ROS.

**Figure 2:** Effect of ROS on migration and invasion capacity of subclones and their parental cells by transwell assay. A, SKBR3 subclones migrated faster than parental SKBR3 cells. NAC was able to effectively inhibit the migration of SKBR3 subclones. *P<0.05 vs SKBR3 cells, **P<0.01 vs A clone, #P<0.01 vs B clone (n = 3). B, 4T1 subclones migrated faster than parental 4T1 cells. NAC was able to effectively inhibit the migration of 4T1 subclones. *P<0.05 vs 4T1 cells, **P<0.01 vs C clone, #P<0.01 vs D clones (n = 3).

**Figure 3:** The migration capacity of subclones and their parental cells was measured by wound healing assay. A–B, The subclones migrated faster than the parental cells SKBR3 cells (A) and 4T1 cells (B). NAC was able to effectively inhibit the migration of the subclones.

### Inhibition of ROS Generation Decreased Cell Motility and Invasion

To further confirm whether ROS were increased in subclone cells, we measured the H_2_O_2_ concentrations in these subclones using the commercial assay kit [24]. As expected, we found that H_2_O_2_ was increased in these subclones (data not shown), and NAC significantly inhibited generation of H_2_O_2_ in subclones (Figure 4A). Furthermore, H_2_O_2_ promoted cell migration and invasion, while its scavenger PEG-catalase decreased cell migration and invasion in subclone cells (Figure 4B, 4C, 4D, Figure S3), suggesting that ROS play a role in cell motility and invasion. More importantly, mitochondria-target SOD mimetic, mito-TEMPO [28] inhibited migration and invasion in subclone cells (Figure 4B, 4C, 4D, Figure S3).

**Figure 4:** PEG-catalase and mito-TEMPO inhibited migration and invasion in subclone cells. A, The H_2_O_2_ concentrations were measured in subclone cells treated with NAC. *P<0.01 vs control in A clone, **P<0.01 vs control in B clone, #P<0.01 vs control in C clone, ##P<0.05 vs control in D clones (n = 3). B, Wound healing assay was conducted to measure the migration capacity of A subclone cells treated with 100 µM H_2_O_2_, 200 units/ml PEG-catalase, 25 nM mito-TEMPO, respectively. Images were captured at 24 h after wounding. C, Migration assay was performed in A subclone cells treated with indicated reagents. D, Invasion capacity of A subclone cells treated with indicated reagents was detected by transwell assay.

### ROS Induced HIF-1α and VEGF Expression

Next, we explore the molecular mechanism of ROS-mediated migration and invasion. Since mitochondrial ROS production has been implicated in the stabilization of HIF-1α during hypoxia [20], we measured HIF-1α expression under both hypoxia and normoxia conditions. As cobalt chloride (CoCl_2_) has been accepted as a hypoxic mimetic agent, we used 500 µmol/L CoCl_2_ to treat cells for 30 minutes before the cells were lysed. As shown in Figure 5, the subclones exhibited increased expression of HIF-1α under normoxic and hypoxic conditions. NAC inhibited not only normoxic HIF-1α expression but also hypoxic HIFα expression in both subclones (Figure 5A, 5B). VEGF, a crucial angiogenic factor for controlling angiogenesis and vasculature, is one of the most prominent HIF-1 target genes. Therefore, we further measured VEGF expression in these subclones. We found that these subclones have increased expression of VEGF (Figure 5A, 5B). We also observed that VEGF expression was significantly decreased after NAC treatment in both subclones (Figure 5A, 5B). These results suggest that ROS could induce HIF-1α and consequently leads to increased VEGF expression. To further validate the role of ROS in regulation of HIF-1α, the subclone cells were treated with PEG-calatase and mito-TEMPO, respectively. We observed that H_2_O_2_ upregulated HIF-1α expression, whereas both PEG-calatase and mito-TEMPO down-regulated the expression of HIF-1α in subclone cells (Figure 5C, 5D). Taken together, our findings demonstrated that ROS play a critical role in cell migration and invasion partly through induction of HIF-1α.

**Figure 5:** ROS promoted HIF-1α and VEGF expression in subclone cells. A, ROS led to increased expression of HIF-1α and VEGF in SKBR3 subclones. SKBR3 subclones showed higher normoxic and hypoxic HIF-1α level than the parental SKBR3 cells. VEGF expression was more increased in SKBR3 subclones than in the parental SKBR3 cells. HIF-1α and VEGF expression in SKBR3 subclone were significantly inhibited by NAC. B, ROS led to increased expression of HIF-1α and VEGF in 4T1 subcloneswhereas NAC was able to attenuate the ROS induced expression of HIF-1α and VEGF. C–D, H_2_O_2_ promoted HIF-1α expression, while PEG-catalase and mito-TEMPO inhibited HIF-1α expression in A clone (C) and C clone (D).

### ROS Promoted Cell Motility by Upregulation of HIF-1α Expression

To determine the role of HIF-1α in ROS-mediated cell motility and invasion, we constructed the expression vector of HIF-1α small interfering RNA to silence HIF 1α expression. The constructs were sequenced to confirm that there are no unwanted mutations (Fig. 6A). The interfering effects were determined by Western blotting analysis. HIF-1α protein expression was significantly inhibited by its shRNA transfection (Fig. 6B). Then we measured cell mobility and invasion ability after depletion of HIF-1α. The results indicate that HIF-1α shRNA transfected cells significantly decreased cells mobility and invasive capacity compared to control cells (Fig. 6C, 6D, 6E). Our results suggest that rotenone initially generate mitochondrial dysfunction and increased ROS production which, in turn, affect tumor cell motility and invasive capacity by upregulation of HIF-1α expression.

**Figure 6:** ROS promoted aggressive cellular behaviors by up-regulating HIF-1α expression. A, The sequence of inserts in the shRNA vector clone. B, Cells with HIF-1α shRNA showed decreased HIF-1α expression compared with the control. C, Cells with HIF-1α shRNA showed decreased migration ability compared with the control as documented by transwell migration assay. **P<0.05 vs A clone (n = 3) D, Cells with HIF-1α shRNA showed decreased invasive capacity compared with the control as documented by transwell invasion assay. **P<0.05 vs A clone (n = 3) E, Wound healing assay showed that cells with HIF-1α shRNA migrated slower than the control.

## Discussion

Mitochondria possess many biological functions, including the production of ATP, housing numerous biochemical reactions, generating ROS, and governing apoptosis [29]. Numerous studies have suggested that these mitochondrial processes may play important roles in tumor initiation and progression [30], [31]. For example, mitochondrial ROS have been implicated in malignant cell transformation [32]. Moreover, it has been suggested that mitochondrial ROS may be important in the maintenance of malignant phenotype through regulation of HIF-1α [28]. In this study, we tested the hypothesis that additional mitochondrial alterations acquired after malignant transformation may increase ROS production which will further contribute to cancer development via ROS-dependent HIF-1α and VEGF pathways to promote cancer cell migration and invasion.

To achieve our goal, we choose rotenone to induce mitochondrial dysfunction to investigate whether rotenone could induce ROS production. Both subclones of breast cancer cells showed higher ROS consistent with declined mitochondrial respiration function, as suggested by decreased ATP generation through oxidative phosphorylation, increased ATP generation through glycolysis, higher glucose uptake and lactate production. These subclones also exhibited increased cellular motility and ability to invade through Matrigel. These malignant behaviors were inhibited by the antioxidant NAC, PEG-Calatase, and mito-TEMPO, indicating the important role of ROS, which is associated with mitochondrial dysfunction.

Although some researchers investigated the role of ROS in carcinogenesis, the exact mechanisms how ROS are involved in tumorigenesis are unclear. Recently, a number of studies have suggested that mitochondrial ROS are involved in the stabilization and activation of HIF under hypoxic conditions [21]. It is known that HIF-1α, which is induced by hypoxia, growth factors, and oncogenes, plays a pivotal role in tumor growth and angiogenesis [13]. ROS affect HIF-1α expression under gastric ischemic conditions, suggesting that ROS can regulate HIF-1α expression in gastric ischemia [33]. Moreover, increased ROS and ROS-dependent stabilization of HIF under conditions of normal oxygen tension have also been reported in cancer cells by suppression of SdhB expression [20]. Furthermore, Xia et al. found that the stabilization of HIF-1α via ROS generation led to the binding of HIF-1α to the FoxM1 promoter, resulting in increased FoxM1 oncoprotein expression in hepatocellular carcinoma [34]. Recently, mitochondria-target antioxidant mito-TEMPO has been demonstrated to inhibit redox-dependent HIF-1α-mediated cancer pro-survival signaling pathways [28]. Consistent with these reports, our results clearly suggest that increased ROS production is required for HIF-1α stabilization in the mitochondrial dysfunction cells induced by rotenone, and these effects were attenuated by antioxidant NAC, PEG-Calatase, and mito-TEMPO. Therefore, our study indicates that ROS promote breast cancer progression, which is in part mediated through up-regulation of HIF-1α expression in breast cancer cells.

Multiple studies have demonstrated that ROS regulate VEGF expression in various human cancers [35]. For example, Xia et al. reported that ROS regulate angiogenesis and tumor growth, which is mediated through upregulation of VEGF [36]. Moreover, Liu et al. found that ROS up-regulate VEGF and HIF-1α through the activation of Akt and p70S6K in human cancer cells [37]. Interestingly, HIF-1α has been found to control VEGF in a variety of human cancer cells [38], [39]. Notably, HIF-1α-mediated up-regulation of VEGF is important in the switch to the angiogenic phenotype during early tumorigenesis [40]. Therefore, these findings suggest that ROS govern VEGF production which is in part mediated through up-regulation of HIF-1α. In line with these reports, we revealed that high levels of ROS production caused elevated VEGF expression by regulating HIF-1α. Conversely, the decrease of HIF-1α expression by ROS inhibitors suppressed VEGF transcriptional activation. Taken together, our present study suggests that mitochondrial dysfunction in breast cancer cells with high ROS production promotes cell mobility and invasion which is in part mediated through HIF-1α and VEGF. However, further in-depth investigation is warranted to explore the molecular insight into the role of ROS-mediated tumorigenesis *in vivo*.

## Supporting Information

Figure S1 **ROS were measured in subclones by DCF-DA method.** A–B, comparison of ROS generation by parental SKBR3 cells (A) and 4T1 cells (B), and their subclones as assessed by using CM-H2DCF-DA measurement done by flow cytometry.
(TIF)

Figure S2 **Effect of ROS on migration and invasion capacity of subclones and their parental cells by transwell assay.** A, The invasive capacity of SKBR3 subclones was higher than the parental SKBR3 cells and was effectively inhibited by NAC. B, The invasive capacity of 4T1 subclones was higher than the parental 4T1 cells and was effectively inhibited by NAC.
(TIF)

Figure S3 **PEG-catalase and mito-TEMPO inhibited migration and invasion in C subclone cells.** A, The migration capacity of C subclone cells treated with different reagents was measured by wound healing assay. B, Migration assay was performed in C subclone cells treated with indicated reagents. C, Invasion capacity of C subclone cells treated with indicated reagents was detected by transwell assay.
(TIF)
